The article "Contribution of α,β-Amyrenone to the Anti-Inflammatory and Antihypersensitivity Effects of Aleurites moluccana (L.) Willd" was published in 2014. Journal: Biomed Res Int.

# Contribution of *α*,*β*-Amyrenone to the Anti-Inflammatory and Antihypersensitivity Effects of *Aleurites moluccana* (L.) Willd.

**DOI:** 10.1155/2014/636839

**Published:** 2014-10-19

**Authors:** Nara Lins Meira Quintão, Lilian W. Rocha, Gislaine Franciele Silva, Simone Reichert, Vanessa D. Claudino, Ruth Meri Lucinda-Silva, Angela Malheiros, Márcia Maria De Souza, Valdir Cechinel Filho, Tania M. Bellé Bresolin, Marina da Silva Machado, Theodoro Marcel Wagner, Christiane Meyre-Silva

**Affiliations:** ^1^Universidade do Vale do Itajaí (UNIVALI), Centro de Ciências da Saúde, Rua Uruguai, No. 458, 88302-202 Itajaí, SC, Brazil; ^2^Núcleo de Investigações Químico-Farmacêuticas (NIQFAR) da Universidade do Vale do Itajaí (UNIVALI), Rua Uruguai, No. 458, 88 302-202 Itajaí, SC, Brazil

## Abstract

The aim of the study was to analyze the constituents of the dichloromethane fraction obtained from* A. moluccana* and also to evaluate the anti-inflammatory and antinociceptive properties of *α*,*β*-amyrenone isolated from* A. moluccana* in mice. The dichloromethane fraction was evaluated by gas chromatography and submitted to purification. The mixture of *α*,*β*-amyrenone was isolated and then evaluated using the carrageenan-induced paw-oedema or pleurisy and CFA-induced arthritis models in mice. Five triterpenes, *α*,*β*-amyrenone, glutinol, and *α*,*β*-amyrin were isolated from dichloromethane fraction of* A. moluccana* leaf extract. The mixture of *α*,*β*-amyrenone, dosed orally, was able to reduce mechanical hypersensitivity and paw-oedema induced by carrageenan, interfering with neutrophil migration. Similar results were observed in the carrageenan-induced pleurisy model. Repeated administration of the compounds was also effective in reducing the mechanical sensitization and oedema developed in the arthritis model induced by CFA. In conclusion, the results demonstrate that *α*,*β*-amyrenone interferes in both acute and chronic inflammatory processes. We can infer that these effects involve, at least in part, a reduction in the neutrophil migration. Therefore, it seems reasonable to suggest that *α*,*β*-amyrenone could represent a new therapeutic tool for the management of painful and inflammatory diseases, especially those presenting a chronic profile.

## 1. Introduction

Analgesic drugs used to treat acute and long-lasting pain have been found to be only partially effective and are commonly associated with side effects that hamper their long-term use [1]. Currently, natural products, particularly medicinal plants, have attracted great interest in the pharmaceutical industry, with the aim of obtaining an effective, safe, and accessible therapy for patients.

*Aleurites moluccana* (L.) Willd., belonging to the Euphorbiaceae family, is commonly known as “Candlenut tree” or “Indian walnut.” Widely distributed in the south and southeast of Brazil, the leaves are used in folk medicine to treat fever, inflammation, asthma, hepatitis, headache, gastric ulcer, and other ailments. Its seeds are used as an antirheumatic and as a fertilizer [2, 3].

In a previous study, the hydroalcoholic extract of* A. moluccana* leaves has been demonstrated to remarkably reduce the nociception in mice, and the flavonoid swertisin 2′′-*O*-rhamnosyl, isolated from ethyl acetate fraction, is partially responsible for this activity [4, 5]. Further* in vivo *antinociceptive assays have led to an emphasis on the analgesic effect of the standardized dried extract of* A. moluccana* with 3% of flavonoid 2′′-*O*-rhamnosyl swertisin, the compound used as chemistry marker of this species. This flavonoid exhibited antinociceptive effect by interacting with opioid, dopaminergic, and oxidonitrergic system [6, 7]. These results support the development of a new herbal medicine for painful processes, as proposed in the patent already granted [8].

Examining the dichloromethane fraction from the leaves, we identified other compounds that may contribute to the activities mentioned above. Among some known compounds, the presence of the triterpenes mixture of *α*,*β*-amyrenone (Figure 1) was identified. Triterpenes are compounds with anti-inflammatory and analgesic effect reported by several researchers and are present in plants used in folk medicine in inflammatory and painful processes [9, 10]. Triterpenes as ursolic acid, lupeol, *α*,*β*-amyrin, and others have proven effects [10–12]. Concerning *α*,*β*-amyrenone, the anti-inflammatory and antinociceptive effects of these compounds particularly against models of inflammation and chronic pain have been little studied. Thus, the present study aimed to evaluate the anti-inflammatory and anti-hypersensitivity effects of *α*,*β*-amyrenone using different models of inflammation and hypersensitivity in mice.

## 2. Materials and Methods

### 2.1. Drugs and Reagents

The following drugs and reagents were used: *β*-amyrin (Fluka, 12777305 32806083), *λ*-carrageenan (Fluka Riedel-de Haën, Seelze, Germany); CFA, EDTA, HTAB, hydrogen peroxide and TMB (Sigma Aldrich Co., St. Louis, MO, USA); Evans blue dye, Türk solution and May-Grünwald-Giemsa dye, NaCl, and NaPO_4_ (Merck, Brazil); Heparin (LIQUEMINE, Roche, Brazil); 0.9% NaCl solution (different commercial sources); retention index mixture of linear hydrocarbons for GC (Sigma Chemical Company, St. Louis, USA). All drugs were diluted in 0.9% NaCl solution.

### 2.2. Plant Material and Extraction

*Aleurites moluccana* L. Willd. was collected in June 2010 in Tijucas, SC, Brazil, and a voucher specimen was deposited at the herbarium Barbosa Rodrigues (BRH, Itajaí, SC, Brazil) under number VCFilho001. The leaves of the dried plant (5 kg) were extracted with methanol at room temperature for 7 days. After this period, the solution was evaporated in vacuum to obtain methanol crude extract, with a yield of 246.5 g (4.93%). Liquid-liquid partitioning was performed on the extract dissolved in 30% H_2_O in ethanol using dichloromethane and ethyl acetate. The fractions were filtered and concentrated using a rotary evaporator and then evaporated to dryness. The yields of the dichloromethane and ethyl acetate fractions obtained were 28.5% and 18.3%, respectively.

### 2.3. Purification of Dichloromethane Fraction

Part of dichloromethane fraction (66.38 g) was submitted to purification using column chromatography (*θ*i 5.4 cm), packed with silica gel (820 g), and eluted with* n*-hexane (Hex) gradually enriched with ethyl acetate (AcOEt) and ethanol. Fifty-two fractions of 200 mL each were collected. The fraction 9–40 (18.72 g) was submitted to column chromatography (*θ*i 3.5 cm), packed with silica gel (276 g), eluted with hexane and gradually enriched with ethyl acetate and ethanol. Thirty-five subfractions of 25 mL each were collected. From the subfraction 7-8, eluted with hexane : ethyl acetate 95 : 5, a mixture of *α*,*β*-amyrenone was obtained giving a yield of 100 mg. Glutinol was obtained from the subfraction 9-10 [elution solvent Hex-AcOEt (95 : 5)] giving a yield of 51 mg. The mixture of *α*,*β*-amyrin was obtained from the subfraction 11-12, elution solvent Hex-AcOEt (90 : 10) giving a yield of 1.170 g and from subfraction 15, friedelenol (61.8 mg) was obtained.

### 2.4. Gas Chromatography (GC)

The dichloromethane fraction was directly analyzed by gas chromatography with electron impact ionization (70 eV) coupled with a GC2010 (Shimadzu, Kyoto, Japan, model GCMS-QP2010S). The column used was 100% methyl silicone DB-1 (30 m × 0.25 mm × 0.25 *μ*m), supplied by Agilent Technologies J&W. The sample was injected using the split mode (split ratio 1 : 10), with injector temperature and GC-MS interface temperature, both at 300°C. The column temperature was programmed from 220°C (1 min), at 30°C/min to 270°C, then raised to 300°C at a rate of 25°C/min, and held at 310°C for 15 min at a rate of 20°C/min. Helium was used as carrier gas. The MS scan range was 30 to 450 a.m.u. The data were processed and the identification of the components was performed by matching their recorded mass spectra with the standard mass spectra from the National Institute of Standards and Technology (NIST 8.0) libraries data, provided by the software of the GC-MS system and literature data.

### 2.5. Animals

Male and female Swiss mice (25–30 g) obtained from the Universidade do Vale do Itajaí (UNIVALI, Itajaí, Brazil) were used in this study. The animals were housed under optimum conditions of light, temperature, and humidity (12 h light-dark cycle, 22 ± 1°C, 60 to 80% humidity), with food and water provided* ad libitum*. All procedures used in the present study followed the “Principles of Laboratory Animal Care” of NIH publication number 85-23 and were approved by the Animal Ethics Committee of UNIVALI (Protocol numbers 416/2008 UNIVALI). The number of animals (5–8 per group) and the intensity of noxious stimuli used were the minimum necessary to demonstrate consistent effects.

### 2.6. Carrageenan-Induced Mechanical Hypersensitivity

Mice received an i.d. injection of 50 *μ*L of carrageenan (300 *μ*g/paw) under the surface of the right hindpaw [6]. To assess the systemic effect of the drug treatment, the mice were previously dosed orally with *α*,*β*-amyrenone (23.5 *μ*mol/kg), indomethacin (27.9 *μ*mol/kg), or vehicle (10 mL/kg, 0.9% NaCl solution), 1 h before carrageenan injection. The mechanical hypersensitivity of all the groups was assessed by means of Von Frey hair (VFH), for up to 24 h after carrageenan administration, as described below.

### 2.7. Carrageenan-Induced Paw Oedema

The animals were pretreated orally with *α*,*β*-amyrenone, dissolved in Tween 0.5% and saline, (23.5 *μ*mol/kg), indomethacin (27.9 *μ*mol/kg), or vehicle (10 mL/kg, 0.9% NaCl solution), and, after 1 h, they received a 50 *μ*L i.d. injection in one hindpaw (right paw) of saline 0.9% containing carrageenan (300 *μ*g/paw). The contralateral hindpaw (left paw) received 50 *μ*L of saline and was used as control [13]. Paw oedema was measured using a plethysmometer (Ugo Basile) at different time points after carrageenan injection and was expressed in *μ*L as the difference between the right and left paws.

### 2.8. Complete Freund Adjuvant- (CFA-) Induced Arthritis

The adjuvant-induced arthritis model used in the present study was similar to that described by Schiene et al. [14] with minor modifications. The animals received in the right hindpaw an i.d. injection of 50 *μ*L of a emulsion containing CFA (1 mg/mL; heat-killed and dried* Mycobacterium tuberculosis*, each milliliter of vehicle containing 0.85 mL paraffin oil plus 0.15 mL mannide monooleate) mixed with saline (1 : 1 oil/saline). As a control, the contralateral paw (left paw) received 50 *μ*L of saline. The animals were orally pretreated with *α*,*β*-amyrenone (2.35–23.5 *μ*mol/kg) or vehicle (10 mL/kg, 0.9% NaCl solution), twice a day, for 8 days, starting at the 14th day of CFA injection, until the 22nd day. Dexamethasone (1.27 *μ*mol/kg) was dosed once every 2 days. The mechanical hypersensitivity of left-end right hindpaw of all the groups was assessed by means of Von Frey hair (VFH), and the paw oedema was measured using a plethysmometer (Ugo Basile) at several time points following CFA injection.

### 2.9. Induction of Pleurisy and Measurement of the Appraised Parameters

The experiments were carried out according to the methodology described by Da Silva Buss et al. [15]. To evaluate the exudation into the pleural cavity, animals received an Evans blue dye solution (25 mg/kg, 0.2 mL, i.v.) and, after 24 h, the animals were orally pretreated with *α*,*β*-amyrenone (23.5 *μ*mol/kg), indomethacin (27.9 *μ*mol/kg), or vehicle (10 mL/kg, 0.9% NaCl solution). After 1 h, they were lightly anaesthetized with ether, and carrageenan (1 mg/cavity, 0.1 mL) was injected into the right pleural cavity. The animals were sacrificed 4 h after the carrageenan injection and the thorax was immediately opened. The pleural cavity was washed with 1 mL of saline (NaCl 0.9%) plus heparin (20 IU/mL), and the exudate was collected. Instead of carrageenan, control animals received sterile saline solution (0.1 mL) in the pleural cavity. Total cell counts were performed in Neubauer chambers by means of an optical microscope, after diluting a sample of the fluid collected from the pleural space with Türk solution (1 : 40). Cellular smears were prepared with an aliquot (0.1 mL) of pleural lavage to determine the differential leukocyte count. The slides were stained with May-Grünwald-Giemsa dye and observed under immersion objective. Another sample of the pleural fluid (0.5 mL) was used to indirectly determine the exudation, through the concentration of Evans blue dye. The amount of dye was estimated at 600 nm by interpolation from a standard curve constructed for Evans blue in the range of 0.5–25 *μ*g/mL.

### 2.10. Von Frey Hairs-Induced Hindpaw Withdrawal Response

The procedures were performed as described by Quintão et al. [16]. To evaluate mechanical hypersensitivity, the mice were placed individually in clear Plexiglas boxes (9 × 7 × 11 cm) on elevated wire mesh platforms, to allow access to the ventral surface of the right hindpaw. The withdrawal response frequency was measured following 10 applications (duration of 1 s each) of Von Frey hairs (VFH, Stoelting, Chicago, IL, USA). The stimuli were delivered from below, to the plantar surface of the right hindpaw. The animals were acclimatized for 30 min before behavioural testing. A VFH of 0.6 g produces a mean withdrawal frequency of about 15%, which is considered to be an adequate value for the measurement of mechanical. Therefore, 0.6 g VFH was used throughout this study. To determine the basal mechanical thresholds, all the groups were evaluated 24 h before the test. For comparison, in the results of experiments, we consider this measure as time zero, before the animals receiving induction with CFA or carrageenan.

### 2.11. Myeloperoxidase (MPO) Activity

Neutrophil recruitment to the mouse paw was indirectly assessed by measuring tissue myeloperoxidase (MPO) activity, as described previously [17]. For this purpose, animals were treated with *α*,*β*-amyrenone (23.5 *μ*mol/kg) or vehicle (10 mL/kg, p.o.) and, after 1 h, they received a 50 *μ*L i.d. injection of carrageenan (300 *μ*g/paw) into the right hindpaw. Saline injected paws were used as a control. Animals were sacrificed 6 h after the application of carrageenan. The subcutaneous tissue of the paws was removed, homogenised at 5% (w/v) in EDTA/NaCl buffer (pH 4.7), and centrifuged at 10,000 rpm for 15 min at 4°C. The pellet was resuspended in 0.5% hexadecyltrimethylammonium bromide buffer (HTAB; pH 5.4), and the samples were frozen and thawed three times in liquid nitrogen. Upon thawing, the samples were recentrifuged (10,000 rpm, 15 min, 4°C), and 25 *μ*L of the supernatant was used for the MPO assay. The enzymatic reaction was assessed with 1.6 mM tetramethylbenzidine (TMB), 80 mM NaPO_4_, and 0.3 mM hydrogen peroxide. The absorbance was measured at 650 nm, and the results were expressed as optic density (OD) per milligram of tissue.

### 2.12. Statistical Analysis

The results are presented as the mean ± SEM of 5 to 8 animals. The percentages of inhibition were calculated using the entire time course of each experiment and reported as the mean ± SEM of inhibitions obtained for each individual experiment at the 4th and 24th hours. Statistical comparison of the data was performed by two-way analysis of variance (ANOVA) followed by Bonferroni's posttest or one-way ANOVA followed by Dunnett's posttest. *P* values lower than 0.05 (*P* < 0.05 or less) were considered significant.

## 3. Results

### 3.1. Phytochemical Analyses

Phytochemical analyses with dichloromethane fraction from* Aleurites moluccana* leaves led to the isolation of triterpenes, a mixture of *α*,*β*-amyrenone (**1**), glutinol (**2**), a mixture of *α*,*β*-amyrin (**3**), and friedelenol (**4**) yields 2.5 × 10^−3^, 1.3 × 10^−3^, 3 × 10^−2^, and 1.5 × 10^−3^% calculated in relation to dry plant. The compounds were identified using spectral data (^1^H and ^13^C-NMR) compared with those previously reported in the literature [4, 18].

*α*,*β*-Amyrenone (**1**). Amorphous white solid. ^13^C NMR data (CDCl_3_, 75.5 MHz): *δ*39.4 (C1), 34.7 (C2), 217.3 (C3), 47.4 (C4), 55.3 (C5), 19.6 (C6), 32.5 (7), 39.3 (C8), 46.7 (C9), 36.6 (C10), 23.5 (C11), 124.1 (12), 139.7 (13), 42.0 (C14), 28.8 (C15), 26.1 (C16), 33.7/32.4 (C17), 59.1/47.3 (C18), 39.6/46.9 (C19), 39.5/31.2 (C20), 34.7 (C21), 37.1/41.5 (C22), 25.6 (C23), 21.5 (C24), 15.4 (C25), 16.7 (C26), 23.5/25.9 (C27), 28.1 (C28), 17.5/33.3 (C29), 21.4/23.6 (C30). EIMS:* m/z*: 424 [M]^+^, 409, 218, 203, 189, 161, 135, 122, 95, 81, 69, 55.

*α*,*β*-Amyrin (**1**). Amorphous white solid. ^13^C  NMR data (CDCl_3_, 75.5 MHz): *δ*38.7 (C1), 27.3 (C2), 78.3/79.0 (C3), 38.8 (C4), 55.3 (C5), 18.3/8.5 (C6), 32.8 (7), 40.0/38.8 (C8), 47.7 (C9), 36.9/37.6 (C10), 23.0 (C11), 124.3/121.8 (12), 139.3/145.1 (13), 41.8 (C14), 28.7/26.2 (C15), 27.0 (C16), 33.7/32.5 (C17), 58.9/47.4 (C18), 39.6/46.9 (C19), 39.6/31.1 (C20), 31.2/34.8 (C21), 41.5/37.2 (C22), 28.2 (C23), 15.5 (C24), 15.6 (C25), 16.9 (C26), 23.3/26.0 (C27), 28.4 (C28), 17.4/33.3 (C29), 21.3/23.7 (C30). EIMS:* m/z*: 426 [M]^+^, 409, 218, 203, 189, 161, 135, 122, 95, 81, 69, 55.

### 3.2. Gas Chromatography (GC) Analyses

The chromatogram of the dichloromethane fraction (Figure 2) revealed the presence of main eight substances with a retention time of 9.323, 9.589, 9.741, 9.950, 10.024, 10.731, 11.227, and 11.461 minutes, identified on the chromatogram as 1 to 8, and attributed to the compounds *β*-amyrenone, *β*-amyrin, *α*-amyrenone, glutinol, *α*-amyrin, unknown, friedelenol, and friedelenone, respectively, when compared with the MS database and the literature [19].

### 3.3. Pharmacological Results

The results presented in Figure 3 demonstrated that i.d. injection of carrageenan into the mice hindpaw induces a prominent reduction in mechanical withdrawal threshold (*P* < 0.001). The systemic treatment of mice with *α*,*β*-amyrenone (23.5 *μ*mol/kg, p.o.), 1 h before the carrageenan injection, was able to significantly reduce the hypersensitivity. Indomethacin (27.9 *μ*mol/kg), used as positive control for this experiment, also inhibited the mechanical hypersensitivity induced by carrageenan for up to 24 h (two-way ANOVA, *F* = 30.52, df = 5, and *P* < 0.0001 for time and *F* = 94.86, df = 2, and *P* < 0.0001 for treatment). Mice treated with *α*,*β*-amyrenone or indomethacin, at the same doses mentioned above, also presented inhibition of hindpaw oedema when compared with vehicle treated group (two-way ANOVA, *F* = 4.61, df = 3, and *P* = 0.005 for time and *F* = 63.13, df = 2, and *P* < 0.0001 for treatment; Figure 4).

It is well established that CFA injection into the rat hindpaw induces prominent paw oedema, which is observed as early as 2 h afterwards and persists for up to 28 h. The assessment of CFA-induced oedema and mechanical hypersensitivity in the advanced phases (14 days before CFA injection) is widely adopted as an arthritis model [20]. In this study, mechanical hypersensitivity was significantly reduced in mice pretreated with *α*,*β*-amyrenone (2.35–23.58 *μ*mol/kg, p.o.) or dexamethasone (1.27 *μ*mol/kg, s.c.), when compared with animals treated with vehicle or vehicle (10 mL/kg, o.p.) (Figure 5(a). Two-way ANOVA, *F* = 23.71, df = 6, and *P* = 0.0001 for time and *F* = 289.3, df = 5, and *P* < 0.0001 for treatment), when compared with the group treated with vehicle. Similar results were obtained in the evaluation of the left hindpaw (Figure 5(b); two-way ANOVA, *F* = 7.69, df = 6, *P* = 0.0001 for time, and *F* = 67.79, df= 5, *P* < 0.0001 for treatment). The same treatments were able to significantly reduce long-term oedema caused by CFA (Figure 5(c); two-way ANOVA, *F* = 3.66, df = 7, and *P* = 0.0001 for time and *F* = 235.3, df = 5, and *P* = 0.0008 for treatment).

In another set of experiments, the anti-inflammatory effect of *α*,*β*-amyrenone (23.5 *μ*mol/kg, p.o.) was evaluated using the carrageenan-induced pleurisy model in mice. Intrapleural injection of carrageenan induces a marked inflammatory response in the mouse pleural cavity, characterized by neutrophil migration and plasma exudation at 4 h. In the present study, oral treatment with *α*,*β*-amyrenone (23.5 *μ*mol/kg, p.o.), given 1 h prior to pleurisy induction, produced a significant decrease in cellular migration to the pleural cavity (Figure 6(a); one-way ANOVA, *F* = 22.11, df = 3, and *P* < 0.0001), mainly by inhibiting the neutrophils influx (Figure 6(b); one-way ANOVA, *F* = 40.33, df = 3, and *P* < 0.0001). However, *α*,*β*-amyrenone treatment did not significantly alter the mononuclear cell migration (Figure 6(c); one-way ANOVA, *F* = 11.44, df = 3, and *P* = 0.0022). A significant reduction was observed regarding the plasma exudation of mice treated orally with *α*,*β*-amyrenone (Figure 6(d); one-Way ANOVA, *F* = 44.45, df = 3, and *P* < 0.0001). Significant inhibition was obtained with mice treated with indomethacin in all the parameters evaluated (Figures 6(a)–6(d)).

The effect of oral treatment with *α*,*β*-amyrenone on paw polymorphonuclear cells infiltration was indirectly assessed by measuring MPO activity (Figure 7). *α*,*β*-Amyrenone was capable of significantly inhibiting MPO activity at all the concentrations tested, when compared with mice treated with vehicle (one-way ANOVA, *F* = 21.89, df = 5, and *P* < 0.0001).

## 4. Discussion

Studies conducted by our research group have already demonstrated the antinociceptive activity of* A. moluccana* dried extract [4, 6, 7]. Such promising results prompted us to investigate the main components of this plant. The use of chromatographic procedures with* A. moluccana* leaves led to the isolation and identification of triterpenes: mixture of *α*,*β*-amyrenone (**1**), glutinol (**2**), and mixture of *α*,*β*-amyrin (**3**). The *α*-amyrin triterpene has a basic skeleton of the ursane type and the *β*-amyrin triterpene has a basic skeleton of the oleanane type, with the only difference between them being the methyl position on the E-ring. The EIMS showed that the molecular peak in M^+∙^ 424 corresponding to mixture of *α*,*β*-amyrenone and M^+∙^ 426 to *α*,b-amyrin and both compounds have base peak at* m/z* = 218. The peaks 218, 203, and 189 are characteristic of fragmentation retro Diels-Alder type of the ring C typical of olean-12-enes and ursan-12-enes.

In order to identify the presence of the mixture of *α*-amyrenone and *β*-amyrenone (**1**) and their ratio in the dichloromethane fraction, this fraction was analyzed by GC. As Figure 2 shows, eight peaks were detected by GC and identified as *β*-amyrenone, *β*-amyrin, *α*-amyrenone, glutinol, *α*-amyrin, friedelenol, and friedelenone, respectively, by comparing their MS spectra with those of the MS database. It was also observed that the ratio of *α* to *β*-amyrenone was 57.3 : 42.7 and the ratio of *α* to *β*-amyrin was 45.9 : 54.1. These values were confirmed by integration of olefins hydrogen in both mixtures of compounds by H^1^NMR analysis.

In the present study, various pharmacological models of inflammation and pain were used in order to find out if *α*,*β*-amyrenone could also be one of the constituents of* A. moluccana *responsible for the pharmacological effect. Due to the small amount isolated, and the pilots trials performed in our laboratories, the compounds were evaluated pharmacologically in single dose. In the first set of experiments, we analyzed the antihypersensitive and anti-inflammatory effects using carrageenan-induced hyperalgesia and paw oedema models in mice [16, 21]. Our study demonstrated that oral treatment reduced the mechanical hypersensitivity induced by carrageenan in mice. This effect was the greatest in the first hour after carrageenan injection, and persisted for up to 6 h after injection. Interestingly, the effect observed with the mixed compound was similar to that observed in animals treated with indomethacin, but with a more prolonged effect (for up to 24 h). Was also observed in the present study *α*,*β*-amyrenone, when dosed orally, was capable of reducing paw oedema induced by carrageenan injection, similar to the effect of indomethacin, demonstrating that the anti-hypersensitivity effects are due, at least in part, to the anti-inflammatory effects.

When injected into the plantar surface of the animal's hindpaw, carrageenan causes inflammation (with characteristic oedema) which results in hyperalgesia [22]. The carrageenan-induced paw edema test is a highly reproducible and well-researched model for evaluating the acute anti-inflammatory actions of natural products.

It is well established through tests that tissue injury resulting from the injection of carrageenan causes the release of different chemical mediators, including prostaglandin E2 (PGE_2_) [23], mast cell products [24], neuropeptides [25], and cytokines such as tumor necrosis factor-alpha (TNF*α*) and interleukin 1-beta (IL-1*β*) [26].

To obtain new results on the anti-inflammatory effect of *α*,*β*-amyrenone, another classic model of inflammation was used: carrageenan-induced pleurisy. The model involves the participation of several cell types and mediators [27]. The mouse pleural inflammatory response induced by carrageenan constitutes an inflammatory model characterized by two distinct phases: (1) 4 h after carrageenan injection and (2) 48 h after carrageenan injection. The first phase is marked by leukocyte recruitment, predominantly neutrophils, and plasma leakage into the pleural cavity. The second phase is marked by an increase in mononuclear cells and greater exudation, compared with the first phase [28]. Myeloperoxidase, adenosine-deaminase, and products of pathways that are stimulated by nitric oxide synthase (iNOS) have been implicated in several aspects of the inflammatory cascade in this model including plasma exudation and cell migration. In this context, Saleh et al. [29] previously demonstrated in this same model of inflammation that MPO activity and nitrate/nitrite (NO) levels significantly increase 4 h after carrageenan-induction of inflammation in the mouse model of pleurisy. In our study, the parameters considered were cell migration and plasma exudation into the pleural cavity at 4 h after intrapleural carrageenan injection. As expected, we evidenced marked accumulation of pleural exudate followed by an intense migration of inflammatory cells to the pleural cavity after pleural carrageenan injection and mice treated orally with *α*,*β*-amyrenone presented a significant reduction in accumulated pleural exudates. Moreover, inhibition of polymorphonuclear cell migration was observed, although this was not effective in decreasing the number of mononuclear cells in the pleural cavity. It is important to mention that similar results were obtained with the positive control, indomethacin. The ability of *α*,*β*-amyrenone to reduce the migration of leukocytes, particularly neutrophils, was confirmed even if indirectly by the reduction in MPO activity. As reported [30], MPO is a common* in vivo *index of neutrophil infiltration and inflammation, as well as a marker of oxidative stress. Results demonstrated that *α*,*β*-amyrenone markedly suppressed MPO activity in inflamed tissues of animal paws, with s indicating that both oxidative stress might be alleviated with the treatment of *α*,*β*-amyrenone. Therefore, another possible mechanism behind the anti-inflammatory effect could be attributed to its antioxidative activity.

Cunha et al. [31] have suggested that the release of primary mediators responsible for carrageenan-induced mechanical hypersensitivity is preceded by the production of a cascade of proinflammatory cytokines. Likewise, neutrophil migration appears to represent a pivotal step in this cascade of events evoked by carrageenan [32]. Additionally, it is important to mention that the hypersensitivity induced by carrageenan injection is directly correlated with the production of the cytokine IL-1*β* and the CXC chemokine CINC-1 [33], contributing to the inflammatory process. Indeed, there is convincing and recent evidence indicating the relevance of neutrophil migration in pain processing mechanisms [32, 34]. In fact, we are not able to precisely conclude as to the mechanisms involved in the antihypersensitive and anti-inflammatory effects of *α*,*β*-amyrenone, but they appear to be dependent on its ability to inhibit neutrophil migration.

The effect of *α*,*β*-amyrenone on inflammatory hypersensitivity induced by i.d. injection of CFA was also investigated in this study. The inflammation induced by CFA develops rapidly and may persist for several weeks or months. The hypersensitivity is mediated by local sensitization of nociceptors and involves immune response and changes in the central nervous system [35]. Surprisingly, repeated treatment completely abolished the mechanical hypersensitivity induced by CFA injection. Furthermore, mice treated with *α*,*β*-amyrenone presented a significant reduction in paw volume. Similar results were obtained with the corticoid dexamethasone.

As previously reported in this study, together *α*,*β*-amyrenone, *α*-amyrin, glutinol, *β*-amyrin, friedelenol friedelenone, and swertisin 2′′-*O*-rhamnosyl, are part of the chemical composition* A. moluccana.* Some of these compounds exhibit antinociceptive and anti-inflammatory effect and may also be associated with anti-inflammatory and analgesic properties of the plant. A special emphasis should be given regarding the pharmacological effects of *α*-amyrin and *β*-amyrin. In fact, the activity of *α*-amyrin and *β*-amyrin, alone or mixed, is well documented in the literature. In experiments conducted in our laboratories, Meyre-Silva et al. [4] demonstrate that the mixture of *α*-amyrin and *β*-amyrin is capable of inhibiting the abdominal writhing induced by acetic acid in mice. Otuki et al. [36] also reported dose-dependent antinociceptive activity of the mixture of these compounds when dosed systemically, spinally, and supraspinally, and it seems to interfere with the protein kinase C (PKC) and protein kinase A-sensitive pathways. The anti-inflammatory effects of *α*-amyrin were also investigated by Medeiros et al. (2007) [37], providing* in vivo* evidence that *α*-amyrin exhibits strong and rapid onset of topical anti-inflammatory actions in mouse TPA-induced ear oedema, involving, at least in part, the reduction of PKC*α* and mitogen activated protein kinases (MAPKs) activation and inhibition of nuclear factor kappa-light-chain-enhancer of activated B cells (NF-*κ*B) activity that culminated in a reduction in PGE_2_ levels, through the inhibition of the cyclooxygenase-2 (COX-2) expression. Recently, Simão da Silva et al. [38] demonstrated that the antihyperalgesic and anti-inflammatory effects of the mixture *α*,*β*-amyrin depend on its ability to bind to the cannabinoid receptors CB_1_ and CB_2_, reduce the release of cytokines (TNF*α*, IL-1*β*, IL-6, and KC), and inhibit the activation of transcriptional factors (NF-*κ*B and CREB).

Soldi et al. [39] revealed that modifications to *α*,*β*-amyrin could alter its efficacy and potency. For example, the oxidation of hydroxyl group present in carbon 3 giving rise to *α*,*β*-amyrenone decreases in potency when evaluated by the acetic acid model. On the other hand, in our study, it was observed that the activity of this compound was similar to that of *α*,*β*-amyrin.

In fact, although the dry plant extract studied also contain the compounds already mentioned above in this work, we show that *α*-*β*-amyrinone can also act against the painful and inflammatory processes. Before this study, the antinociceptive activity of *α*,*β*-amyrinone had not been investigate.

In summary, our results demonstrate that *α*,*β*-amyrenone interferes in both acute and chronic inflammatory process. We can infer that these effects involve, at least in part, a reduction in neutrophil migration. Therefore, it seems reasonable to suggest that *α*,*β*-amyrenone could represent a new therapeutic tool for the management of painful and inflammatory diseases, especially those presenting a chronic profile. Experiments are in progress to evaluate the molecular mechanism through which this active compound exerts its effect.

## Figures and Tables

**Figure 1:** *α*,*β*-Amyrenone isolated from* Aleurites moluccana* leaves.

**Figure 2:** Chromatogram of dichloromethane fraction from* Aleurites moluccana* leaves.

**Figure 3:** Effects of oral treatment with *α*,*β*-amyrenone (23.5 *μ*mol/kg), indomethacin (27.9 *μ*mol/kg), or vehicle (10 mL/kg, 0.9% NaCl solution) on mechanical hypersensitivity induced by i.d. injection of carrageenan (300 *μ*g/paw) in mice. Each group represents the mean of 5 to 8 animals, and the vertical lines indicate the SEM. Significantly different from control values: ^**^ *P* < 0.01 and ^***^ *P* < 0.001. Two-way ANOVA followed by Bonferroni's post hoc test.

**Figure 4:** Effects of oral treatment with *α*,*β*-amyrenone (23.5 *μ*mol/kg), indomethacin (27.9 *μ*mol/kg), or vehicle (10 mL/kg, 0.9% NaCl solution), on paw oedema induced by i.d. injection of carrageenan (300 *μ*g/paw) in mice. Zero (time zero) corresponds to baseline measurement of animals performed 24 hours before the test. Each group represents the mean of 5 to 8 animals, and the vertical lines indicate the SEM. Significantly different from control values: ^*^ *P* < 0.05, ^**^ *P* < 0.01, and ^***^ *P* < 0.001. Two-way ANOVA followed by Bonferroni's post hoc test.

**Figure 5:** Effect of the treatment with *α*,*β*-amyrenone (7.07–70.7 *μ*mol/kg, p.o.), dexamethasone (1.27 *μ*mol/kg, s.c), or vehicle (10 mL/kg, 0.9% NaCl solution, p.o.) on the mechanical hypersensitivity of the (a) right and (b) left hindpaw and paw oedema induced by i.d. injection of CFA (50 *μ*L/paw; 1 : 1 0.9% NaCl solution) into the mice right hindpaw. Zero (day zero) corresponds to baseline measurement of animals performed 24 hours before the test. Each group represents the mean of 5 to 8 animals, and the vertical lines indicate the SEM. Significantly different from saline group values ^#^ *P* < 0.001, and significantly different from control values ^*^ *P* < 0.05, ^**^ *P* < 0.01, and ^***^ *P* < 0.001. Two-way ANOVA followed by Bonferroni's post hoc test.

**Figure 6:** Effect of *α*,*β*-amyrenone (23.5 *μ*mol/kg), indomethacin (27.9 *μ*mol/kg), or vehicle (10 mL/kg, 0.9% NaCl solution), dosed orally, on pleurisy induced by carrageenan (1 mg/cavity, 4 h). (a) Total cells. (b) Mononuclear cells. (c) Neutrophils. (d) Evans blue content (exudation). Each column represents the mean of 6 to 10 animals and the vertical bars represent the SEM. Significantly different when compared with group injected with carrageenan and treated with vehicle (^***^ *P* < 0.001) and saline injected group (^#^ *P* < 0.01). One-way ANOVA followed by Dunnett's post hoc test.

**Figure 7:** Effect of oral treatment with *α*,*β*-amyrenone (7.07–70.7 *μ*mol/kg) or vehicle (10 mL/kg, 0.9% NaCl solution) on the increase in MPO activity induced by i.d. injection of carrageenan (300 *μ*g/paw) into the mice hindpaw. Each group represents the mean of 3 to 4 animals, and the vertical lines indicate the SEM. Significantly different from saline group values ^#^ *P* < 0.001, and significantly different from control values ^**^ *P* < 0.01. One-way ANOVA followed by Dunnett's post hoc test. Control group (C), naïve group (N), saline injected group (S).
